# Polymorphisms in the *TNFA and IL6* Genes Represent Risk Factors for Autoimmune Thyroid Disease

**DOI:** 10.1371/journal.pone.0105492

**Published:** 2014-08-15

**Authors:** Cecília Durães, Carla S. Moreira, Inês Alvelos, Adélia Mendes, Liliana R. Santos, José Carlos Machado, Miguel Melo, César Esteves, Celestino Neves, Manuel Sobrinho-Simões, Paula Soares

**Affiliations:** 1 Institute of Molecular Pathology and Immunology of the University of Porto (IPATIMUP), Porto, Portugal; 2 Faculty of Medicine of the University of Porto, Porto, Portugal; 3 Faculty of Medicine of the University of Coimbra, Coimbra, Portugal; 4 Department of Endocrinology, Diabetes and Metabolism, University and Hospital Center of Coimbra, Coimbra, Portugal; 5 Unit of Endocrinology, Faculty of Medicine, University of Coimbra, Coimbra, Portugal; 6 Department of Endocrinology, Hospital of S. João, Porto, Portugal; 7 Department of Pathology and Oncology, Faculty of Medicine of the University of Porto, Porto, Portugal; Instituto de Higiene e Medicina Tropical, Portugal

## Abstract

**Background:**

Autoimmune thyroid disease (AITD) comprises diseases including Hashimoto's thyroiditis and Graves' disease, both characterized by reactivity to autoantigens causing, respectively, inflammatory destruction and autoimmune stimulation of the thyroid-stimulating hormone receptor. AITD is the most common thyroid disease and the leading form of autoimmune disease in women. Cytokines are key regulators of the immune and inflammatory responses; therefore, genetic variants at cytokine-encoding genes are potential risk factors for AITD.

**Methods:**

Polymorphisms in the *IL6*-174 G/C (rs1800795), *TNFA*-308 G/A (rs1800629), *IL1B*-511 C/T (rs16944), and *IFNGR1*-56 T/C (rs2234711) genes were assessed in a case-control study comprising 420 Hashimoto's thyroiditis patients, 111 Graves' disease patients and 735 unrelated controls from Portugal. Genetic variants were discriminated by real-time PCR using TaqMan SNP genotyping assays.

**Results:**

A significant association was found between the allele A in *TNFA*-308 G/A and Hashimoto's thyroiditis, both in the dominant (OR = 1.82, CI = 1.37–2.43, *p-value* = 4.4×10^−5^) and log-additive (OR = 1.64, CI = 1.28–2.10, *p-value* = 8.2×10^−5^) models. The allele C in *IL6*-174 G/C is also associated with Hashimoto's thyroiditis, however, only retained significance after multiple testing correction in the log-additive model (OR = 1.28, CI = 1.06–1.54, *p-value* = 8.9×10^−3^). The group with Graves' disease also registered a higher frequency of the allele A in *TNFA*-308 G/A compared with controls both in the dominant (OR = 1.85, CI = 1.19–2.87, *p-value* = 7.0×10^−3^) and log-additive (OR = 1.69, CI = 1.17–2.44, *p-value* = 6.6×10^−3^) models. The risk for Hashimoto's thyroiditis and Graves' disease increases with the number of risk alleles (OR for two risk alleles is, respectively, 2.27 and 2.59).

**Conclusions:**

This study reports significant associations of genetic variants in *TNFA* and *IL6* with the risk for AITD, highlighting the relevance of polymorphisms in inflammation-related genes in the etiopathogenesis of AITD.

## Introduction

Autoimmune diseases, which affect 5 to 7% of the population and are frequently responsible for severe disability, represent a major cause of chronic illness and an important issue in general healthcare [1]. Autoimmune thyroid diseases (AITD), including Hashimoto's thyroiditis (HT) and Graves' disease (GD), are the most common organ specific autoimmune disorders [2].

HT and GD stand for the major portion of clinical presentations in a wide range of thyroid autoimmune conditions, which culminate in thyroid dysfunction [3]. HT is a T cell-mediated organ-specific autoimmune disease characterized by lymphocytic infiltration that leads to thyroid cells loss, clinically expressed by hypothyroidism [4]. In contrast, GD patients exhibit hyperthyroidism, which is due to excessive secretion of the thyroid hormone induced by specific autoantibodies to the thyrotropin receptor (TSHR) produced by TSHR-reactive B cells [5].

The etiology of HT and GD involves common as well as unique pathways. Both diseases carry thyroid reactive T cells that escape the tolerance process and infiltrate the thyroid. Nevertheless, distinct pathways lead thyroid-reactive T cells to either cause the death of thyroid cells in HT or their stimulation in GD [6]. Thus, there is presently awareness that the genetic susceptibility to HT and GD involves both shared and unique genes [7].

Several factors, including genetic, hormonal, environmental, and nutritional elements are involved in the initiation and/or development of AITD, however the pathophysiologic changes seen in AITD are mediated by inflammatory cytokines [3]. IL1β, IL6 and TNFα cytokines, and IFNGR1 have proinflammatory activity and represent important facilitators of the immunologic process involved in HT and GD as components of the autoimmune response [8]–[14]. Various cytokines and respective genetic polymorphisms have been reported to be associated with AITD, yet the results are inconsistent [8]–[12], [15].

In the present work, a case-control study was performed to assess if the risk to develop HT and GD is associated with the promoter single nucleotide polymorphisms (SNPs) *IL1B*-511 C/T (rs16944), *TNFA*-308 G/A (rs1800629), *IL6*-174 G/C (rs1800795), and *IFNGR1*-56 T/C (rs2234711). This study reports significant associations of promoter SNPs in *TNFA* and *IL6* with the risk for AITD and the combined effect of risk variants for HT and GD development.

## Materials and Methods

### Study population

A total of 1266 Portuguese subjects were included in the study. The patients group comprised 531 individuals (mean age 45.4±16.0 years), 111 diagnosed with GD and 420 diagnosed with HT. Patients were enrolled in the study from 2007 until 2013 and the number obtained reflects the relative incidence reported for the two diseases (1GD/3.8HT) [16]. Patients' clinicopathological details are described in Table 1. The diagnosis of GD was established on the basis of clinical findings, decreased serum thyroid stimulating hormone (TSH) (<0.35 IU/mL), elevated serum free thyroxine (FT4) (>1.48 ng/dL) and/or free triidothyronine (FT3) (>3.71 pg/mL), positive serum antibodies to TSH-receptor (TRAb) (>1.8 IU/L), and typical ultrasound signs (hypoechogenicity and high perfusion). Diagnosis of HT was obtained based on clinical findings, positive serum antibodies to thyroid peroxidase (TPOAb) and/or thyroglobulin (TgAb) (according to the method applied before or after March 2009 in the Department of Clinical Pathology of Hospital S. João), and characteristic ultrasound signs (hypoechogenicity and non-homogeneous texture).

**Table 1:** Demographic data and clinical characteristics of patients with Graves' disease and Hashimoto's thyroiditis.

		Gender	Age of diagnosis	Free T3	Free T4	TSH	TgAb positive	TPOAb positive	TRAb positive
Patients groups		(F:M)	(y)	(pg/mL)	(ng/dL)	(IU/L)	n (%)^a^	n (%)^a^	n (%)^b^
Graves' disease	n	95∶16	111	89	91	109	108	110	83
		6∶1	44.47±16.11	3.86±2.67	1.67±1.74	1.38±4.49	98 (88.3)	91 (82.7)	34 (41.0)
Hashimoto's thyroiditis	n	385∶35	420	418	420	393	410	411	404
		11∶1	45.6±15.95	3.00±1.26	1.36±1.49	2.34±3.78	368 (89.8)	298 (72.5)	54 (13.4)

Abbreviations: F, female; M, male; y, years. Data are expressed as mean ± standard deviation. **n** indicates the number of patients from whom we obtained clinical data and was different for each characteristic.

a Until March 2009 the Siemens ADVIA Centaur CP immunoassay system was the applied assay for thyroid function tests (reference values: antithyroglobulin 0.0–0.60 IU/mL and antithyroid peroxidase 0.0–60.0 IU/mL); after that the laboratory changed to Abbot Architect i2000 (reference values: antithyroglobulin <4.11 IU/mL and antithyroid peroxidase <5.61 IU/mL). For this reason only quantitative assessment (positive/negative) was considered.

b Positive serum TRAbs (>1.8 IU/L). All HT patients were submitted to thyroid hormone replacement therapy (levothyroxine).

The control group included 735 unmatched samples obtained from unrelated healthy blood donors (mean age 49.2±16.8 years). This group consisted of permanent residents in the catchment area of Hospital of S. João (Porto, Portugal), selected during the assembling of the EpiPorto cohort [17]. Enrollment of participants was performed under approval of Hospital of S. João ethic committee and included written informed consent for data and DNA usage.

### SNP genotyping

Patients and controls genomic DNA was isolated from blood using standard proteinase K digestion with phenol/chloroform extraction. SNPs *IL1B*-511 C/T (rs16944), *TNFA*-308 G/A (rs1800629), *IL6*-174 G/C (rs1800795), and *IFNGR1*-56 T/C (rs2234711) were genotyped using TaqMan Pre-Designed SNP Genotyping Assays (Applied Biosystems, Carlsbad, USA). PCR amplification and allelic discrimination were performed according to product specifications with the ABI 7500 Fast real-time PCR system (Applied Biosystems, Carlsbad, USA). Optimization of each TaqMan Assay was performed using controls of known genotype selected through DNA sequencing. Cases and controls were randomized during genotyping and 5% of the samples were genotyped in duplicate to assess the genotyping error rate (genotype concordance was 100%).

### Statistical analysis

Genotype frequencies of all SNPs were obtained using SPSS 21 (IBM SPSS Statistics). Compliance of alleles at individual *loci* with the Hardy-Weinberg equilibrium was measured at the level of the control population using a χ^2^ test (level of significance set to *p-value* <0.05) implemented in the SNPassoc 1.6-0 package in R [18].

Comparison of genotype frequencies between groups defined by *status* (HT and GD patients *versus* controls) was assessed by unconditional logistic regression (level of significance set to *p-value* <0.05) with the SNPassoc package implemented in R [18] and included gender and age. Odds ratios (OR) with respective confidence intervals (95% CI) were calculated considering the genotypic, dominant and log-additive (per allele) models of inheritance. The adjustment for multiple testing was performed by the false discovery rate (FDR) method [19].

## Results

In the control group, the frequencies of all SNPs did not deviate significantly from those expected under Hardy-Weinberg equilibrium (*p-value* for *IL1B*-511, *TNFA*-308, *IL6*-174 and *IFNGR1*-56 is, respectively, 0.059, 0.122, 0.491 and 0.347). The genotyping success rate of all SNPs was 100% in the control and GD groups and >99% in the HT group. The frequency of genotypes and association parameters are summarized in Table 2.

**Table 2:** Genotypic frequencies and association given by the odds ratio (OR) and 95% confidence intervals (95% CI) between genetic variants in *IL1B*, *TNFA*, *IL6*, and *IFNGR1*, and Graves' disease and Hashimoto's thyroiditis.

	Controls	Graves'disease^a^			Hashimoto's thyroiditis^a^		
Locus/genotype	n (%)	n (%)	OR (95% CI)^b^	*p-value* b	n (%)	OR (95% CI)^b^	*p-value* b
***IL1B*** **-511 C/T**	n = 735	n = 111			n = 417		
CC	327 (44.5)	44 (39.6)	1.00^c^		177 (42.4)	1.00^c^	
CT	309 (42.0)	47 (42.3)	1.04 (0.66–1.63)	0.8775	173 (41.5)	1.00 (0.76–1.32)	0.9984
TT	99 (13.5)	20 (18.0)	1.30 (0.72–2.36)	0.3842	67 (16.1)	1.15 (0.79–1.69)	0.4875
T *carrier vs* CC	408 (55.5)/327 (44.5)	67 (60.4)/44 (39.6)	1.10 (0.73–1.67)	0.6488	240 (57.6)/177 (42.4)	1.04 (0.80–1.34)	0.7910
log-additive (C/T)	963 (65.5)/507 (35.5)	135 (60.8)/87 (39.2)	1.12 (0.84–1.49)	0.4453	527 (63.2)/307 (36.8)	1.05 (0.88–1.26)	0.5766
***TNFA*** **-308 G/A**	n = 735	n = 111			n = 416		
GG	562 (76.5)	72 (64.9)	1.00^c^		277 (66.6)	1.00^c^	
GA	156 (21.2)	34 (30.6)	1.79 (1.13–2.83)	0.0127	123 (29.6)	**1.81 (1.34–2.45)**	**1.2×10^−4^**
AA	17 (2.3)	5 (4.5)	2.43 (0.83–7.08)	0.1046	16 (3.8)	1.95 (0.92–4.13)	0.0797
A *carrier vs* GG	173 (23.5)/562 (76.5)	39 (35.1)/72 (64.9)	**1.85 (1.19–2.87)**	**7.0×10^−3^**	139 (33.4)/277 (66.6)	**1.82 (1.37–2.43)**	**4.4×10^−5^**
log-additive (G/A)	1280 (85.1)/190 (14.9)	178 (80.2)/44 (19.8)	**1.69 (1.17–2.44)**	**6.6×10^−3^**	677 (81.4)/155 (18.6)	**1.64 (1.28–2.10)**	**8.2×10^−5^**
***IL6*** **-174 G/C**	n = 735	n = 111			n = 418		
GG	319 (43.4)	37 (33.3)	1.00^c^		156 (37.3)	1.00^c^	
GC	324 (44.1)	61 (55.0)	1.54 (0.99–2.41)	0.0583	189 (45.2)	1.21 (0.92–1.60)	0.1791
CC	92 (12.5)	13 (11.7)	1.14 (0.57–2.27)	0.7158	73 (17.5)	**1.69 (1.15–2.51)**	**8.3×10^−3^**
C *carrier vs* GG	416 (56.6)/319 (43.4)	74 (66.7)/37 (33.3)	1.45 (0.94–2.23)	0.0865	262 (62.7)/156 (37.3)	1.31 (1.01–1.71)	0.0406
log-additive (G/C)	962 (65.4)/508 (35.6)	135 (60.8)/87 (39.2)	1.18 (0.87–1.59)	0.2925	501 (59.9)/335 (40.1)	**1.28 (1.06–1.54)**	**8.9×10^−3^**
***IFNGR1*** **-56 T/C**	n = 735	n = 111			n = 418		
CC	150 (20.4)	15 (13.5)	1.00^c^		75 (17.9)	1.00^c^	
CT	350 (47.6)	58 (52.3)	1.58 (0.85–2.91)	0.1456	204 (48.8)	1.08 (0.76–1.54)	0.6517
TT	235 (32.0)	38 (34.2)	1.55 (0.81–2.96)	0.1830	139 (33.3)	1.09 (0.75–1.58)	0.6490
T *carrier vs* CC	585 (79.56/150 (20.4)	96 (86.5)/15 (13.5)	1.57 (0.87–2.81)	0.1188	343 (82.1)/75 (17.9)	1.09 (0.78–1.51	0.6214
log-additive (C/T)	650 (60.6)/820 (39.4)	88 (39.6)/134 (60.4)	1.19 (0.88–1.59)	0.2577	354 (42.3)/482 (57.7)	1.04 (0.87–1.25)	0.6828

a The number of cases and controls genotyped for each SNP differs according to their genotyping success.

b Values in bold are statistically significant with a *p-value* cutoff = 0.00892 (after FDR correction).

c Reference estimate. All calculations, except for *IFNGR1*, were performed considering the most frequent allele/genotype as reference.

The *TNFA*-308 A allele is significantly associated with HT risk in the log-additive (OR = 1.64, CI = 1.28–2.10, *p-value* = 8.2×10^−5^) and dominant models (OR = 1.82, CI = 1.37–2.43, *p-value* = 4.4×10^−5^). The frequency of the *TNFA*-308 A allele was also higher in GD than in controls in both log-additive and dominant models (OR = 1.69, CI = 1.17–2.44, *p-value* = 6.6×10^−3^ and OR = 1.85, CI = 1.19–2.87, *p-value* = 7.0×10^−3^, respectively).

A significant association was found between the *IL6*-174 allele C and HT risk in the log-additive model (OR = 1.28, CI = 1.06–1.54, *p-value* = 8.9×10^−3^) but did not reach significance for the dominant model (OR = 1.31, CI = 1.01–1.71, *p-value* = 0.0406) after FDR correction (*p-value* <0.0106).

Statistically significant differences were not observed in the frequencies of genotypes and alleles of the *IL1B*-511 C/T, *IL6*-174 C/G and *IFNGR1*-56 T/C polymorphisms between GD patients and controls, and the *IL1B*-511 C/T and *IFNGR1*-56 C/T polymorphisms between HT patients and controls.

The joint effect of genetic polymorphisms was assessed considering the high-risk genotypes *TNFA* A *carrier* and *IL6* C *carrier* (Table 3). The reference group contains no high-risk genotypes, group 1 contains individuals with one of the high-risk genotypes and group 2 contains individuals with two of the high-risk genotypes. Individuals carrying two high-risk genotypes present an increased risk for GD [OR (CI) = 2.59 (1.46–4.59), *p-value* = 1.2×10^−3^] and for HT [OR (CI) = 2.27 (1.53–3.38), *p-value* = 5.4×10^−5^].

**Table 3:** Genetic risk profile for Graves' disease and Hashimoto's thyroiditis including the susceptibility variants at *TNFA* and *IL6* a.

	Graves' disease		Hashimoto's thyroiditis	
Nr of risk genotypes^a^	OR (95% CI)	*p-value*	OR (95% CI)	*p-value*
**0**	1.00^b^		1.00^b^	
				
**1**	1.09 (0.67–1.79)	0.7282	**1.48 (1.10–2.00)**	**0.0106**
				
**2**	**2.59 (1.46–4.59)**	**1.2×10^−3^**	**2.27 (1.53–3.38)**	**5.4×10^−5^**

Note: The number of cases and controls genotyped for each SNP differs according to their genotyping success rates.

a The reference group (0) contains no high-risk genotypes, group 1 contains individuals with one of the high-risk genotypes and group 2 contains individuals with two of the high-risk genotypes.

b Reference estimate. Values in bold are statistically significant with a *p-value* <0.05.

## Discussion

Our results report significant associations of genetic variants in *TNFA* and *IL6* with HT, and in *TNFA* with GD. The risk odds were increased whenever an individual presented more than one high-risk genotype. Genetic variants in proinflammatory cytokine genes can have the potential to alter the regulation of the transcript production or function. Considering the role of proinflammatory cytokines in the pathogenesis of the autoimmune response involved in GD and HT, a change in the function or the quantity of a particular cytokine may lead to the initiation or perpetuation of the inflammatory process. The importance of the IL1β, TNFα, IL6, and IFNGR1 in the immunological response is well established in the literature. Thus, SNPs in these cytokines and receptor may have a role in the susceptibility to HT and GD in which the immune response is a major feature.

TNFα plays an important role in the initiation of an adaptive immune response [3]. TNFα is produced by monocytes, T cells, natural killer cells, and mast cells. It is involved in the up-regulation of the HLA class I, activation of phagocytes, induction of IL1, IL6, and TNFα itself and, synergistically with IFNγ, enhancement of the HLA class II expression [11], [20]–[22]. TNFα mRNA is found in thyroid tissue from patients with GD and HT in higher levels than in healthy subjects [23]. Our study reports a statistically significant association between the *TNFA*-308 allele A both with HT and GD. This is in agreement with previous studies for GD [11], [14], [15], [24]–[28] but not for HT [10], [25], [28]. It has been observed that the *TNFA*-308 A allele is associated with a higher level of the *TNFA* transcript, justified by the greater potency of the promoter region to activate the transcription [29], [30], which suggests that the *TNFA*-308 A allele may have a role in the pathogenesis of the AITD. Nevertheless, conflicting data were reported concerning the genotypic and allelic frequencies of the *TNFA*-308 G/A polymorphism in GD and HT [9], [10], [25], [28], [31], [32]. In fact, a meta-analysis of *TNFA* polymorphisms in GD reported an association of the TNFA-308 SNP in Caucasians but not in Asians [33]. The *TNFA* gene is located in the HLA class III domain of the major histocompatibility complex (MHC) [34]. There are studies showing the genetic contribution of the HLA regions for AITD susceptibility [35]–[38]. The HLA are regions of strong linkage disequilibrium, thus it cannot be ruled out that the association of *TNFA* variants with HT and GD might not be due to polymorphisms within *TNFA* itself, but rather to variation in a linked gene [25], [28].

Polymorphisms in the *IL6* promoter region have been implicated in susceptibility to carotid atherosclerosis [39], multiple myeloma [40], and juvenile chronic arthritis [41]. IL6 is mainly produced by mononuclear phagocytes, under stimulation of IL1, TNF or lipopolysaccharide. IL6, a Th2 cytokine, has been connected with the modulation of thyroid cells function, and its expression in thyrocytes correlated positively with the degree of lymphocyte infiltration in HT [42], [43]. Furthermore, IL6 plays a major role in B cell differentiation and T cell proliferation, and the deregulated production of IL6 and its receptor was related with the pathogenesis of autoimmune diseases by inhibition of autoreactive T cell apoptosis [44]. Our study reports an association of the C allele in *IL6*-174 with the risk to develop HT but not GD. This result is consistent with the lack of association with GD in a Polish [8] and Taiwanese populations [11]. In contrast, two other studies in an Iranian [15] and Turkish [27] populations reported association of the *IL6*-174 SNP with GD, albeit in the latter the association was on the threshold of significance. To the best of our knowledge, there are no reports implying the *IL6*-174 G/C polymorphism in HT susceptibility. Current data suggest that the C allele at the −174 position is responsible for lower expression of IL6, leading to lower IL6 serum levels [45], [46]. Other studies have demonstrated that patients with HT have higher serum levels of IL6, inversely correlated with the thyroid function [45], [47], [48]. Nevertheless, it has been reported that the expression of IL6 occurs in a greater proportion of GD patients than in HT patients, which may correlate with the different lymphoid aggregate in the two AITD [43]. There is no evidence that the *IL6*-174 G/C polymorphism is a causal variant for HT, but our results may contribute to clarify some differences in the pathogenesis of HT and GD.

Polymorphisms in the *IL1* gene have been associated with other autoimmune diseases such as rheumatoid arthritis [49], inflammatory bowel disease [50], and systemic lupus erythematosus [51]. IL1β has pleiotropic effects, can alter cytokine production, cell signaling and migration, [52]. Several studies have reported conflicting results regarding the possible role of *IL1B*-511 C/T polymorphism in AITD. The TT genotype has been described as a protective variant for GD [12], [53], [54], however, other studies did not report any association between this polymorphism and GD or HT [10], [55], [56]. In the present study, we also did not observe a significant association between the *IL1B*-511 C/T polymorphism and GD or HT. In agreement with our results, a recent meta-analysis has reported that the *IL1B*-511 SNP is associated with GD in Asians but not in Caucasians [57].

*IFNGR1* encodes a class II cytokine receptor which is ubiquitously expressed in nucleated cells and is the receptor for IFNγ, one of the most important Th1-related cytokines [58]. Several functions have been attributed to IFNγ, such as the enhancement of the expression of the HLA class I, class II and some adhesion molecules on thyrocytes, including intercellular adhesion molecule 1 (ICAM1) and lymphocyte function-associated antigen 3 (LFA3) [15]. Previous studies have proposed a possible association between polymorphisms in IFNγ encoding genes and the autoimmune response in GD [15], [59]. Furthermore, a recent study demonstrated that IFNγR knockout mice remained thyroiditis resistant even after Treg-depletion [60]. In our study, there was no association between the *IFNGR1*-56 T/C polymorphism and both HT and GD.

The association results obtained after *TNFA* and *IL6* genotypes combination reveal a risk increase for individuals harboring more than one high-risk allele/genotype for both HT and GD. These results are compatible with the individual effect of each variant and point to a cumulative effect in the susceptibility for the disease. However, larger studies are necessary to verify these observations since, due to limited statistical power of the GD cohorts especially after genotype combination, one should be cautious when interpreting the results.

It is assumed that multiple factors interfere in the susceptibility and initiation of AITD while others are responsible for the perpetuation of the autoimmune process. Our study contributes to the understanding of individual susceptibility to AITD when *carrier* of risk alleles in certain cytokine-encoding genes (*TNFA* and *IL6*), highlighting the relevance of polymorphisms in inflammation-related genes as molecular markers for AITD.
